# Characterization of Retained Austenite in Advanced High-Strength Steel

**DOI:** 10.1155/2023/9565903

**Published:** 2023-04-17

**Authors:** Shouhua Li, Kejian Li, Longzhu Zhang, Yi Feng, Ziquan Liu, Pengjun Cao, Bo Liu, Jiling Dong

**Affiliations:** ^1^HBIS Hansteel Technology Center, Handan, Hebei 056015, China; ^2^School of Metallurgy and Materials Engineering, Chongqing University of Science & Technology, Chongqing 401331, China; ^3^College of Materials Science and Engineering, Chongqing University, Chongqing 400044, China; ^4^China Automotive Engineering Research Institute Co., Ltd., Chongqing 401122, China; ^5^School of Mechanical Engineering, University of Science and Technology Beijing, Beijing 100083, China

## Abstract

The retained austenite (RA) in advanced high-strength steels directly affects their plasticity. It is very important for the accurate characterization of their content and types. This paper prepared three specimens with three different Mn contents (1.0%, 1.4%, and 1.7%) that are used to obtain high-strength steel by ultrafast cooling heat treatment. The volume content and distribution of the RA were analysed by an X-ray Debye ring measurement system, electron backscatter diffraction (EBSD), and transmission electron microscopy (TEM). In addition, the mechanical tensile test provided the tensile properties and elongation of three specimens. It was finally concluded that when the content of Mn increased, the island-type and thin film-type RA both increased, which may effectively improve the plasticity of the martensitic steels.

## 1. Introduction

The plasticity and toughness of a material bring high profile because the toughness refers to the energy absorbed during stress to fracture. The greater the energy consumed to make materials fracture, the better their toughness. Consuming energy means performing work on the material outside the system. That is, force and displacement (deformation) are required [1]. The ability to withstand stress is characterized by the strength and the ability to deform by plasticity. Thus, the ductile materials have good plasticity [2]. From an engineering point of view, the strength of a material refers to its yield strength. In general, the higher the strength of the material, the higher its plastic deformation resistance and hardness. The toughness is a comprehensive index that reflects the strength and plasticity of materials. More precisely, materials with good toughness have higher strength and better plasticity, which results in higher yield strength and ductility. The preparation of materials with both high strength and good plasticity is the pursuit of the engineering field [3, 4]. The traditional approaches for improving the performance of the martensitic steel include increasing the carbon content, adding a lot of alloying elements such as Cr and Ni, and using the cyclic quenching technology, which makes the steel more expensive and decreases its welding ability. The technology of microstructure control by special rolling and cooling, such as retained austenite (RA) controlling, can be economic and effectively improve the performance of steels [5–7].

The advanced high-strength steel has been widely used in the industrial field due to its good mechanical properties and very high corrosion resistance for structural applications, such as the automobile, transport, and petrochemical industries [8]. However, the RA in steels has been widely studied to further improve the performance and application value of the materials [9]. In general, austenite is soft, which reduces its strength, hardness, and wear-resisting performance, causing the dimensional deformation of its precision parts [10]. Therefore, it is desirable to limit the RA content as much as possible during material production. In martensitic high-strength steels, practical and theoretical studies have shown that in many cases, RA does not damage the properties of steel but effectively improves the plasticity of the material [11].

It has been demonstrated that AISI 4340 has higher fracture toughness after high-temperature quenching. Lai [12] compared the microstructure and properties of the 4340 steel after two different heat treatments. The first one consists in heating the material to 870°C for oil quenching, while the second one consists in heating it to 1200°C and then cooling it to 870°C. The first method contains very little RA, while the second has a large amount of RA film between the martensite lath with a thickness in the range of 10-20 nm. The second process increases the fracture toughness by almost 80%. On the one hand, the toughness level increases due to the martensite morphology changes and the disappearance of the twinned martensite. On the other hand, martensite lath in thin film surrounds the RA, which improves the toughness of the material. Therefore, the RA is effective for improving the toughness of the material.

The RA function in steel grades varies. Existing studies demonstrated that austenite has strong toughness and hydrogen storage capacity. However, the diffuse rate of hydrogen in austenite is much less than that in martensite or ferrite. At room temperature, the diffusion coefficients of hydrogen in low alloy martensite steel and austenite stainless steel are 3.7 × 10^−11^ m^2^/s and 2 ~ 7 × 10^−16^ m^2^/s, respectively. In fact, the interface of the RA and martensite matrix is a strong hydrogen trap. Therefore, an appropriate amount of RA can make good hydrogen traps, which improves the hydrogen embrittlement (HE) resistance of the ultra-high-strength martensitic steels [13–15].

To understand this pattern, this paper focuses on the volume content and distribution of RA in advanced high-strength steel. X-ray Debye ring measurement system [16], electron backscatter diffraction (EBSD), transmission electron microscopy (TEM), and mechanical tensile test were used for the characterization of the RA-contained test specimens.

## 2. Materials and Methods

In this study, three kinds of specimens with increasing Mn content were prepared. The chemical composition of the second one (Mn-1.4%) is similar to that of the commercial steel grade of 1500 MPa. The first and third schemes have higher (1.7%) and lower (1.0%) Mn, respectively. Steel smelting was performed using a 50 kg laboratory melting furnace. The chemical compositions of the ingot specimens are shown in Table 1.

Figure 1 shows the heat treatment process of the three specimens, which is detailed as follows:

1. The ingot was hot rolled to a 20 mm thick plate. The plates were then sheared and homogenized at 1250°C for 2 h. The plates were hot rolled to 3.5 mm. The finishing rolling temperature was almost 900°C
2. The hot bands were held in a furnace at 620°C for 1 h, followed by air cooling to simulate the industrial coiling process
3. The hot bands were ground to remove the decarburized layers and cold-rolled to a thickness of 1 mm
4. The annealing consisted of heating the specimens to 900°C, isothermal holding for 100 s, cooling to 880°C, and holding for 40 s, followed by quenching in inorganic salt solution
5. Finally, the specimens were tempered at 200°C for 100 s and air-cooled to room temperature

X-ray Debye ring measurement of RA was performed using the *μ*-X360s, which is an X-ray residual stress measurement system (Cr target, Ver. 3.0, Pulstec Industrial Co., Ltd.). This measurement consists in averaging the full ring (500 orientation outputs at one measurement). Microstructural characterization was conducted by scanning electron microscopy (SEM, JEOL-7800) and EBSD (EDAX-TSL). TEM measurements were also performed using a JEOL-2100F operating at 200 kV. For EBSD and TEM observations, thin samples were prepared by cutting cross-sections of the steel plates, mechanical polishing, and double jet electropolishing of the steel substrate (Struers TenuPol-5). The electropolishing was performed with a 90% CH_3_COOH+10% HClO_3_ electrolyte.

## 3. Results

### 3.1. X-Ray Debye Ring Measurement of RA

Figure 2(a) shows two peaks of diffracted X-ray used to calculate the RA. The X-ray diffracted from CrK_*α*_ was 2*θ* of martensite (or ferrite) *α*′ (211) at 156.4° and 2*θ* of austenite *γ* (220) at 128.8°. The Debye ring of two peaks is shown in Figure 2(b). The ideal integrated intensity was then calculated. The equation in Figure 2(c) was used to calculate the integrated intensity ratio per *α* degree. The integrated intensity ratio (*I*_*γ*_) and volume ratio (*V*_*γ*_) are then measured, as shown in Figure 2(d). However, the measurement result can only be used for the relative comparison because it is difficult to calculate the absolute value using this method. The RA was calculated by converting the integrated intensity to the volume of the material.

A Debye ring is formed by diffraction of an X-ray beam on the surface of a polycrystalline metal [16]. Thus, the Debye ring contains information on the state of the surface and the crystals. The average value of the whole Debye ring (*α* degree: 0-360 degree) is the final result. For this measurement, it is necessary to set the sensor unit angle (X-ray incidence angle) and height (sample distance) to detect the diffraction from austenite (128.8*°*) inside a 2D detector according to the following condition.

Figure 3 shows the raw data sampling of Debye ring of the 1.0 Mn specimen. More precisely, Figures 3(a)–3(f) present the Debye ring in 2D, the Debye ring in 3D, the distortion image, 2D extraction, 3D extraction, and profile analysis.

Figure 4 shows the corresponding RA measurement result: from (a) to (c), the Debye ring, peak strength, and *γ*Ri. It can be deduced that the RA of the 1%, 1.4%, and 1.7% Mn specimens were 0.5%, 0.9%, and 3.5%, respectively. The repeated tests proved that the data stability was greater than 90%.

### 3.2. EBSD Analysis of RA

Figure 5 shows the EBSD phase mapping of the tested specimens, where the green color represents martensite and the red color represents RA. The areas of the three mapping images are the same, and the number and area fraction are gradually increasing function of the RA. The calculation results show that the area proportions of red pixels in the 1%, 1.4%, and 1.7% Mn specimens are 0.44%, 0.77%, and 3.12%, respectively.

Figure 6 shows higher magnification EBSD analysis of the 1.7% Mn content specimen: from (a) to (c), the image quality of the martensite structure, the inverse pole figure of crystal orientations, and the phase mapping with added high-angle grain boundaries. Lots of fine grains were found in the interstitial position of the martensite lath. The phase scanning results show that part of the very fine grains is the RA. In addition, all the apparent RA are located along with the high-angle grain boundaries.

### 3.3. TEM Analysis of RA

Figure 7(a) shows a TEM bright-field image of the martensite and RA structure of 1.7% Mn content specimens, and Figures 7(b) and 7(c) present selected areas of the electron diffraction patterns (SADPs) corresponding to the B and C red circles in Figure 7(a). The analyses of SADPs show that zone B is austenite and zone C is martensite. Therefore, region B is identified as RA with a size of almost 500 nm.

Figure 8 shows TEM images of the martensite lath of the 1.7% Mn content specimens. The bright-field image on a standard fine martensite lath is shown in Figure 8(a), and the lath thickness is in the range of 200-400 nm. The SADPs are inside the image, which forms the corresponding circular region. The SADP proved that the crystal zone axis of the martensite lath is [110]. The high-resolution TEM image of the lath boundary in Figure 8(b) shows that the thickness of the intermediate region is approximately 7 nm. The simulative diffraction patterns and inverse Fourier transform are calculated on the images marked by red squares. The results are highlighted by red and blue borders, respectively. The diffraction pattern analysis proved that the *γ*-Fe phase is inside the intermediate region and the martensite structure is on both sides. In addition, the orientation relationship of the selected electron diffractions is proved as [111] *α*′//[110]_*γ*_. This corresponds to the Kurdjumov-Sachs (K-S) relationship between austenite and martensite [17, 18]. Therefore, the RA is in the form of thin film type in the presence of fine grains (similar to the island type).

The engineering stress-strain diagram of the three test specimens is shown in Figure 9. The 1%, 1.4%, and 1.7% Mn specimens have maximum tensile strengths of 1479 MPa, 1502 MPa, and 1512 MPa, respectively. Their yield strengths are 1170 MPa, 1194 MPa, and 1248 MPa, while their total elongations are 5.9%, 6.7%, and 6.9%, respectively. It can be seen from the tensile results that when the Mn content increases, the tensile strength and elongation of the material increase. This is due to the fact that Mn promotes the stability of austenite, which results in the increase of the RA content in the matrix and the improvement of the solid solution strengthening effect of the Mn element. The mechanical properties of the material are also affected by the small changes in the grain size, lath thickness, and dislocation density.

## 4. Discussion

Based on the above test results, the following conclusions can be drawn. The X-ray Debye ring, EBSD, and TEM measurements show that RA should exist in the martensitic steel. In addition, the RA content increases with the increase of the added amount of Mn. Moreover, the RA is island type and thin film type. However, the resolutions of the X-ray, EBSD, and TEM are different. In fact, it is assumed that the X-ray can detect all the types of RA. The step size of EBSD is 100 nm, and thus, it can recognize only the island-shaped RA. The RA types and volume fraction in the three test specimens are summarized in Table 2. The thin film-type RA was calculated as the X-ray measurement result minus the EBSD result, which also increases with the increase of the added amount of Mn.

The mechanical tensile test results confirm that in three kinds of martensite steel, when the Mn content increases, the RA content increases, and the thin film-type RA exists in the interface of martensite lath, which significantly improves the plasticity of the material. However, most of the RA has island type by fine grains, and therefore, the property cannot be improved. The RA between the martensite laths increases the resistance to crack propagation because the toughness level of the material is improved. When the crack encounters RA in the advancing process, a deformation occurs, which increases the energy consumption required by the crack air combat. The RA is prone to slip during deformation, which reduces the stress concentration at the crack tip and thus requires greater stress for crack instability and propagation.

Moreover, the transformation-induced plasticity (TRIP) phenomenon appears in the normal range of crack preface. In addition, due to the existence of RA, the interface of pure body-centered cubic structure is replaced by body-centered cubic and face-centered cubic high lattice planes, which is not conducive to crack propagation [19–21]. However, the above theory only applies when the RA is distributed in the cracks of martensite lath. When the RA exists in the form of a block, the above strengthening mechanism cannot be applied.

Several studies indicated that the RA as island type is the main microstructural constituent controlling this toughness, which highlights the need for a precise identification of these constituents in the studies dealing with the microstructure-toughness relation [22, 23]. In the temperature of ferrite nucleation, the carbons will diffuse in the austenite. Near the interface of austenite and ferrite, high concentrations of carbon from austenite to carbon-rich austenite island form. With the quick cooling process, austenite evolves into martensite [24]. The martensite-austenite island is then generated, as shown in Figure 7. The refined heterogeneous phase unit enhances the ductility in quenched ultra-high-strength steels for the fine austenite. The strengthening mechanism is similar to the precipitation strengthening and pinning dislocation movement [25, 26]. Therefore, RA is as a kind of tough microstructure present in advanced high-strength steel.

The mechanical stability of RA has chemical, size, and shape stabilities. All kinds of advanced high-strength steel containing stable RA will exhibit HE stability. However, the deformation (e.g., tension deformation and deformation induced by applied stress during the part use) can induce RA to undergo martensite transformation, which will reduce the delay fracture resistance [27, 28]. This is due to the hard and brittle martensite transformation of residual austenite induced by deformation, which results in reducing the strength and toughness of the steel. For example, in the manufacturing process of steel parts, RA will undergo martensite transformation under force or strain, leading to the increase of the HE sensitivity [29, 30]. Therefore, the RA control can significantly improve the strength and toughness of the steel and successfully improve the HE resistance.

## 5. Conclusion

In this study, X-ray Debye ring, EBSD, and TEM measurements were used to characterize the RA in three 1500 MPa grade advanced high-strength steels. The X-ray Debye ring and EBSD observations confirmed that the RA content increases with the increase of the added amount of Mn. The TEM observations confirmed that two types of RA (fine grain (island) type with thickness of ~500 nm and thin film type with thickness of ~7 nm) exist between the martensite laths. The results showed that RA increased in both types. The engineering stress-strain diagram of the three test specimens showed that their maximum tensile strengths, yield strengths, and extended rates increase with the increase of the added amount of Mn. Thus, the RA control by Mn addition can effectively improve the strength and toughness of high-strength steels.

## Figures and Tables

**Figure 1:** Diagram of the thermomechanical treatments.

**Figure 2:** (a) X-ray peak, (b) Debye ring, (c) calculation formula, and (d) diffraction intensity with angle.

**Figure 3:** RA measurement: (a) Debye ring in 2D, (b) Debye ring in 3D, (c) distortion, (d) 2D extraction, (e) 3D extraction, and (f) profile.

**Figure 4:** RA measurement: (a) Debye ring, (b) peak strength, and (c) *γRi*.

**Figure 5:** EBSD phase mapping of (a) 1%, (b) 1.4%, and (c) 1.7% Mn content specimens, where the green and red color represent martensite and RA, respectively.

**Figure 6:** EBSD analysis of the (a) image quality, (b) inverse pole figure, and (c) phase mapping with added high-angle grain boundaries.

**Figure 7:** (a) TEM bright-field image of the martensite and RA structure and (b, c) SADPs in the corresponding zones marked in (a).

**Figure 8:** (a) TEM observation on the martensite lath showing the SADP in the corresponding circular region and (b) high-resolution TEM image of the lath boundary showing the *γ*-Fe phase.

**Figure 9:** Engineering stress-strain diagram of the three test specimens.

**Table 1:** Chemical compositions of the test specimens (wt.%).

Specimens	C	Si	Mn	P	S	Fe
1.0% Mn	0.21	0.21	1.00	0.011	0.002	Bal.
1.4% Mn	0.21	0.21	1.40	0.010	0.001	Bal.
1.7% Mn	0.21	0.22	1.70	0.012	0.002	Bal.

**Table 2:** RA types and volume fraction in the three test specimens.

Specimens	Total volume fraction of RA by X-ray measurement	Island-type RA by EBSD measurement	Thin film-type RA by calculation
1% Mn	0.5%	0.44%	0.06%
1.4% Mn	0.9%	0.77%	0.13%
1.7% Mn	3.5%	3.12%	0.38%

## Data Availability

No data were used to support this study.
